# Expression Level, Correlation, and Diagnostic Value of Serum miR-127 in Patients with Acute Respiratory Distress Syndrome

This article has been retracted.

**DOI:** 10.1155/2021/2257764

**Published:** 2021-09-22

**Authors:** Hui Lin, Lingxiang Jiang, Yiqun Ren, Fen Sheng, Luxi Wang, Sujiang Zhang

**Affiliations:** ^**1**^ Department of General Practice, Taizhou First People's Hospital, Taizhou, Zhejiang 318020, China; ^**2**^ Pulmonary and Critical Care Medicine, Taizhou First People's Hospital, Taizhou, Zhejiang 318020, China

## Abstract

**Objective:**

To analyze the expression of miR-127 in the serum of patients with acute respiratory distress syndrome (ARDS) and to explore its correlation with the severity of ARDS patients and its value as a molecular marker for diagnosis of ARDS.

**Methods:**

70 patients with ARDS admitted to our hospital from September 2017 to September 2019 were selected as the observation group, and 60 healthy persons with physical examination were collected as the control group. RT-PCR was used to detect the serum miR-127 levels of all subjects, and the serum miR-127 levels of the observation group and control group were compared. The oxygenation index (PaO_2_/FiO_2_) of ARDS patients was recorded and divided into three subgroups: mild group, moderate group, and severe group. Serum miR-127 levels of patients in the mild group, moderate group, and severe group were compared. Pearson correlation was used to analyze the relationship between serum miR-127 levels and the severity of ARDS patients. The receiver operating characteristic curve (ROC) was drawn, and the area under the ROC curve (AUC) was used to evaluate the diagnostic value of miR-127 in patients with ARDS.

**Results:**

The serum level of miR-127 (10.15 ± 1.03) in the observation group was significantly higher than that in the control group (3.09 ± 0.62). And in the three subgroups of mild, moderate, and severe, the serum miR-127 level in the moderate group (10.43 ± 0.71) and the severe group miR-127 level (11.05 ± 1.26) were significantly higher than those in the mild group level (9.38 ± 1.24). Pearson correlation analysis showed that the serum miR-127 level was negatively correlated with PaO_2_/FiO_2_ (*r* = −0.715, *P* < 0.05), that is, the serum miR-127 level was positively correlated with the severity of ARDS patients. The area under the curve (AUC) of the diagnostic value of serum miR-127 for ARDS was 0.732 (95% CI 0.607–0.858). When the optimal cutoff value was 0.380, the sensitivity was 59.1% and the specificity was 78.6%, which suggested that miR-127 can be used as a marker for ARDS diagnosis.

**Conclusion:**

There is an increase in miR-127 levels in the serum of ARDS patients. The serum miR-127 level is positively correlated with the severity of ARDS. The higher the level of miR-127, the worse the condition of ARDS, which is positively correlated with the severity of the condition. It suggests that the serum miR-127 level is an important indicator for evaluating the severity of ARDS patients. It can be used as a molecular marker for clinical diagnosis of ARDS.

## 1. Introduction

Acute respiratory distress syndrome is a form of acute respiratory failure due to progressive respiratory distress. The clinical manifestations of ARDS are hypoxemia, pulmonary inflammation, and noncardiogenic pulmonary edema. The pathogenesis involves the aggregation and spread of inflammatory cells, the release of inflammatory factors, and alveolar capillary damage [1, 2]. ARDS has many complex causative factors, with a mortality rate of 35%–50%, posing a serious risk to patients' lives and health [3, 4]. In particular, ARDS caused by infectious factors has a rapid onset and rapid progress without intervention and treatment. According to the different oxygenation index, acute lung injury (ALI) is a milder stage. ARDS and ALI, respectively, represent two different stages of the same disease. The early stage of the disease, the milder stage is ALI; the later stage of the disease, the more severe stage is ARDS. In 2012, the definition of ARDS Berlin published by the European Society of Critical Care in JAMA deleted the nomenclature of ALI. Since then, the disease has been collectively referred to as ARDS. Now, the mild ARDS is basically equivalent to the original ALI. At present, the pathogenesis of ARDS is not fully understood, and the therapeutic effect is not satisfactory. The clinical diagnosis of ARDS is mainly made by patient symptoms and signs, primary causative factors, and laboratory and imaging examinations. It lacks relevant specific biomarkers, and therefore, there are problems such as low specificity [5].

microRNAs are a type of noncoding small RNAs whose function is to regulate gene expression at the posttranscriptional level, and most of them play a negative regulatory role. In terms of lung diseases, studies have shown that miRNAs are related to chronic infection with COPD, ARDS, proliferative pulmonary fibrosis, and other diseases. A large number of cell and animal experiments on ARDS have shown that miRNAs expression changes in ARDS models induced by different injury factors, and studies have found their targets and regulatory signal pathways [6]. The human miR-127 gene is located on chromosome 14q32.31, including miR-136, miR-431, miR-432, miR-433, miR-337, and miR-665 miRNA family, located in the imprinted region of D1k/Gtl2, transcribed in the reverse direction. Human miR-127 can express two mature miRNAs, miR-127-3p and miR-127-5p, because of its precursor. Some studies have also shown that the expression of miR-127 is related to signaling pathways such as NF-*κ*B-TNF*α* and other tumor suppressor genes such as SEPT7 and BCL6. At present, various miRNAs such as miR-125b, miR-127, and miR-135b have been confirmed to be upregulated in the serum of ARDS patients, but their expression in the serum and their diagnostic value for ARDS patients are still inconclusive [7, 8]. In this study, we analyzed the correlation between serum miR-127 expression and the severity of ARDS patients admitted to our hospital and evaluated the diagnostic value of miR-127 for ARDS, in order to provide a clinical basis for the diagnosis and treatment of ARDS and to improve the quality of life of patients through early diagnosis and treatment. The specific studies reports are as follows:

## 2. Materials and Methods

### 2.1. General Information

70 patients with ARDS admitted to our hospital from September 2017 to September 2019 were selected as the observation group. The primary diseases of the patients included pulmonary disease in 20 cases, traumatic injury in 16 cases, pancreatitis in 14 cases, peritonitis in 9 cases, sepsis in 7 cases, hemorrhagic shock in 3 cases, and meningitis in 1 case. The inclusion criteria are that all patients meet the diagnostic criteria of ARDS and the new definition of ARDS in Berlin in 2012 [9, 10]. Based on the time of onset, chest imaging, causes of pulmonary edema, and PaO_2_/FiO_2_ changes, the patient was diagnosed with the disease. The time from onset to admission is less than 48 h, and the age is not less than 18 years old. Exclusion criteria: impaired function of other important organs such as the heart and kidney, autoimmune diseases, and psychiatric diseases. Among the 70 patients, 39 were males and 31 were females, aged 21–74 years old, with an average of (49.37 ± 11.64) years old. 60 physically healthy individuals were collected as the control group. All patients and their families were required to sign an informed consent form for treatment.

### 2.2. Sample Collection

Blood was collected from ARDS patients on an empty stomach before the initial treatment after admission, and the blood was taken from the abdomen of the control group. After the blood was placed in an EDTA anticoagulation tube for 30 minutes, it was centrifuged at 2000 r/min for 5 minutes, and the upper serum was separated and stored in a refrigerator at −80°C. The total RNA was extracted according to the serum RNA extraction kit instructions; the miR-127 primer was designed according to the gene sequence of miR-127 in the miRBase database, and U6 was used as the internal reference. Reverse transcription reactions were performed with the corresponding stem-loop primers according to the reverse transcription PCR kit instructions. The reaction conditions were 16°C for 30 min, 42°C for 30 min, and finally 80°C for 5 min. Real-time quantitative PCR was used for predenaturation at 95°C for 5 minutes, followed by 90°C for 15 s, 60°C for 15 s, and 72°C for 1 minute, for a total of 40 cycles. The experimental operation was carried out in strict accordance with the instructions of the corresponding kit. The serum RNA extraction kit and RT-PCR kit were purchased from TAKARA, Japan, and the miR-127 and U6 primers were synthesized by Shanghai Shenggong Biology Company, as given in Table 1.

### 2.3. Research Methods

ResMed VPAP III noninvasive positive pressure ventilation ventilator or Swiss HAMILTON Medical AG invasive ventilator was used to inhale oxygen and monitor patients in the observation group. The values were recorded at fraction of oxygen absorbed (FiO_2_) = 100% and positive end-expiratory pressure (PEEP) ≤ 5 cm H_2_O. ARDS classification: mild, with an oxygenation index (PaO_2_/FiO_2_) value of 201–300 mmHg; moderate, with a PaO_2_/FiO_2_ value of 101–200 mmHg; and severe, with PaO_2_/FiO_2_ ≤ 100 mmHg. The 70 ARDS patients were divided into three subgroups according to the above classification criteria: mild group (29 cases), moderate group (26 cases), and severe group (15 cases). The age, gender, and primary disease of the three groups of patients were balanced and comparable, and the difference was not statistically significant (*P* > 0.05).

### 2.4. Statistical Methods

SPSS 22.0 software was applied for processing. Two-by-two comparisons were analyzed by the *t*-test. Correlation analysis was performed using the Pearson correlation analysis. Subject working characteristic curves (ROC) were plotted, and the area under the ROC curve (AUC) was used to evaluate the diagnostic value of miR-127 in ARDS patients. *P* < 0.05 was considered a statistically significant difference.

## 3. Result

### 3.1. Comparison of Serum miR-127 Levels between the Observation and Control Groups

The results showed that the serum miR-127 level of the observation group (10.15 ± 1.03) was significantly higher than that of the control group (3.09 ± 0.62). The difference was statistically significant (*P* < 0.05), as shown in Figure 1.

### 3.2. Comparison of Serum miR-127 Levels in the Three Subgroups of Light, Moderate, and Severe Observation Groups

The level of serum miR-127 in the moderate group (10.43 ± 0.71) and the level of serum miR-127 in the severe group (11.05 ± 1.26) were significantly higher than the level of serum miR-127 in the mild group (9.38 ± 1.24), and the differences were statistically significant (*P* < 0.05), as shown in Figure 2.

### 3.3. The Relationship between Serum miR-127 Level and the Severity of ARDS Patients

Pearson correlation analysis showed that the serum miR-127 level was negatively correlated with PaO_2_/FiO_2_ (*r* = −0.715, *P* < 0.05), that is, it was positively correlated with the severity of ARDS, as shown in Figure 3.

### 3.4. The Diagnostic Value of Serum miR-127 Level for ARDS

The area under the diagnostic value curve (AUC) of miR-127 for ARDS was 0.732 (95% CI 0.607–0.858). When the best cutoff value was 0.380, the sensitivity was 59.1% and the specificity was 78.6%, as given in Table 2 and Figure 4.

## 4. Discussion

ARDS is a kind of acute lung injury caused by noncardiogenic and exogenous pathogenic factors in the lungs. The pathogenesis is complex, with high morbidity, high mortality, and disability. [11]. The main pathophysiological changes of ARDS are diffuse alveolar capillary injury, lung interstitial and alveolar edema, alveolar surfactant reduction, alveolar hyaline membrane formation, lung volume reduction, lung tissue compliance reduction, and severe ventilation/blood flow ratio imbalance. The typical imaging manifestations are diffuse infiltrates of the lungs, or even “white lungs,” and the clinical manifestations are hypoxemia that is difficult to correct by simply inhaling oxygen. The Berlin Conference of the European Critical Care Society redefines the diagnostic criteria of ARDS, removes the concept of acute lung injury, and classifies it as mild ARDS [12]. The Berlin definition incorporates the onset time (onset within one week) and PEEP level into the evaluation system and grades the severity of ARDS. ARDS is an acute diffuse lung injury, which can be caused by pathogenic factors directly or indirectly through the airway, including shock, trauma, severe infection and sepsis, aspiration, and metabolic diseases; the infection is ARDS, the most common cause. The incidence of ARDS caused by simple bacteremia is not high, and severe sepsis combined with ARDS can be as high as 35%–45%. ARDS caused by infection is more serious, and the mortality rate is higher. In the past 10 years, the mortality rate of severe pneumonia and ARDS caused by the virus is higher. ARDS can lead to respiratory failure and other symptoms in a short period of time, aggravating the original condition of the patient. Once the diagnosis progresses rapidly, the late intervention of ARDS is limited. If not treated timely and effectively, it will cause serious complications and affect the health of patients. Therefore, the early diagnosis of ARDS is always a key and difficult task for clinicians [13]. At present, the mechanism of ARDS is not fully understood, and the treatment effect is not satisfactory. Further research on the detailed mechanism of the occurrence and development of ARDS is of great significance for in-depth understanding of the pathophysiological process of ARDS and finding new treatment methods.

MiRNAs are a type of endogenous noncoding RNA with important regulatory functions, which can form a silent complex with other molecules to regulate the degradation of target gene mRNA or inhibit the progress of translation, thereby realizing the regulation of protein expression and participating in cell activities. Currently, miRNAs are differentially expressed in a variety of lung diseases. Related studies have shown that in acute lung injury, there are differences in miRNA expression in diseased and normal tissues of patients and specific alterations in peripheral blood [14]. In nonsmall cell lung cancer, a variety of miRNAs and circulating miRNAs with high sensitivity and tissue specificity can be used as potential diagnostic and therapeutic biomarkers for patients with nonsmall cell lung cancer [15]. In ARDS, the same specific expression of miRNAs exists and can be used as a specific molecular marker to diagnose patients [16, 17]. The production process of microRNAs is affected by many factors, including ARDS and other inflammatory reactions. The nature of microRNAs is relatively stable, so they are not easy to be degraded. MicroRNAs are widely distributed in blood, tissues, and other specimens; different specimen processing methods will not cause them to be destroyed. The expression of some microRNAs is time-existent and tissue-specific and has effects on the internal and external environments of cells. Signal changes will produce responses, and it is these characteristics that allow microRNAs to be used as biomarkers to reflect different diseases or different stages of the same disease.

At present, a large number of studies have used methods such as real-time fluorescent quantitative PCR and microribonucleic acid chips to discover the ARDS model caused by different cell experiments and different injury factors and the changes in the miRNA expression profile in the alveolar lavage fluid and serum of ARDS patients, as well as their target genes, participate in the regulation of different cell signaling pathways. The expression of microRNAs such as miR-146a, -155, -214, and -145 is upregulated in the mouse ARDS model induced by LPS, and the expression of microRNAs such as miR-16-23a and 181a-125b is downregulated. The target genes of some microRNAs in ARDS and the signal pathways they participate in the regulation have been studied in depth. For example, the role of miR-146a and miR-155 in ARDS has been studied more clearly. In ARDS, the expression of miR-146a and miR-155 was increased, and they acted on IRAK-1/TRAF-6 and Socs1, respectively, and inhibited their expression to promote the ARDS inflammatory response [18, 19]. A large number of similar studies have investigated the role of different microRNAs in ARDS, providing new ideas for the mechanism research, diagnosis, and treatment of ARDS. However, the mechanism of ARDS is complex, and it is far from enough to study the role of microRNAs in ARDS with existing ideas and experimental methods. At present, most of the research on the role of miRNA in ARDS is based on cell experiments and/or animal model research, which is still far from clinical practice. Therefore, miRNA is of great significance in clinical research.

miR-127 has been more studied in tumors, and high expression of miR-127 exists in a variety of malignant tumors such as esophageal squamous carcinoma and lung cancer [20, 21]. In tumor cells, miR-127 promotes epithelial mesenchymal transition of tumor cells by activating various signaling pathways such as NF-*κ*B-TNF*α*, which in turn accelerates tumor cell proliferation, migration, and drug resistance. miR-127 can also directly inhibit the expression of a variety of tumor suppressor genes, such as SEPT7 and BCL6, thereby promoting tumor cell invasion [22, 23]. Guo Lei et al. found high expression of various miRNAs such as miR-30b, miR-99a, and miR-127 in the serum of ARDS patients [24, 25]. To confirm the above research, we collected the serum of patients with ARDS to detect the level of miR-127 and analyzed the relationship between miR-127 and the severity of the disease and its diagnostic value for ARDS. The results of this study showed that the serum miR-127 levels in patients in the observation group (10.15 ± 1.03) were significantly higher than those in the control group (3.09 ± 0.62). And among the three subgroups of patients in the observation group, mild, moderate, and severe, serum miR-127 levels in the moderate group (10.43 ± 0.71) and serum miR-127 levels in the severe group (11.05 ± 1.26) were significantly higher than those in the mild group (9.38 ± 1.24). It is inferred that serum miR-127 levels can be used to assess the severity of disease in ARDS patients.

The Pearson correlation analysis in this study showed that serum miR-127 levels were negatively correlated with PaO_2_/FiO_2_ (*r* = −0.715, *P* < 0.05), that is, positively correlated with the severity of ARDS. The area under the curve (AUC) of the diagnostic value of miR-127 for ARDS was 0.732 (95% CI 0.607–0.858). When the best cutoff value is 0.380, the sensitivity is 59.1% and the specificity is 78.6%, suggesting miR-127 can be used as a new type of molecular marker for the diagnosis of ARDS.

## 5. Conclusion

In conclusion, there is an elevated level of miR-127 in the serum of ARDS patients. The higher the level of miR-127, the more severe the disease of ARDS, which is positively correlated with the severity of the disease, suggesting that the level of serum miR-127 is an important indicator of the severity of the disease in patients with ARDS and can be used as a molecular marker for clinical diagnosis of ARDS.

## Figures and Tables

**Figure 1:** Comparison of serum miR-127 levels between the observation group and control.

**Figure 2:** Comparison of serum miR-127 levels in the three subgroups of light, medium, and severe in the observation group.

**Figure 3:** The relationship between the serum miR-127 level and the severity of ARDS patients.

**Figure 4:** ROC curve of the serum miR-127 level for diagnosis of ARDS.

**Table 1:** miR-127 and U6 PCR primer sequence.

Name	Primer sequence
miR-127	Stem-loop primer (5′-3′): CTCAACTGGTGTCGAGTCGGCAATTCAGTTGAGAGCCAAGC
	Forward primer (5′-3′): AAGGAGCCCCACGAGAAAAA
	Reverse primer (5′-3′): ACCGAACTTGCATTGATTCC

U6	Stem-loop primer (5′-3′): AACGCTTCACGAATTTGCGT
	Forward primer (5′-3′): CTCGCTTCGGCAGCACA
	Reverse primer (5′-3′): AACGCTTCACGAATTTGCGT

**Table 2:** The diagnostic value of the serum miR-127 level for ARDS.

Index	AUC	Asymptotic 95% confidence interval		Best cutoff value	Sensitivity (%)	Specificity (%)
		Lower limit	Upper limit			
miR-127	0.732	0.607	0.858	0.380	59.4	78.6

## Data Availability

The data used and/or analyzed during the current study are available from the corresponding author upon request.
